The article "Estimating the prevalence of food risk increasing behaviours in UK kitchens" was published in 2017. Journal: PLoS One.

# Estimating the prevalence of food risk increasing behaviours in UK kitchens

**DOI:** 10.1371/journal.pone.0175816

**Published:** 2017-06-28

**Authors:** Anna K. Jones, Paul Cross, Michael Burton, Caroline Millman, Sarah J. O’Brien, Dan Rigby

**Affiliations:** 1 Natural Resources Wales, Bangor, United Kingdom; 2 Bangor University, Bangor, Wales, United Kingdom; 3 University of Western Australia, Perth, Australia; 4 University of Manchester, Manchester, United Kingdom; 5 University of Liverpool, Liverpool, United Kingdom; Agricultural University of Athens, GREECE

## Abstract

Foodborne disease poses a serious threat to public health. In the UK, half a million cases are linked to known pathogens and more than half of all outbreaks are associated with catering establishments. The UK Food Standards Agency (FSA) has initiated the UK Food Hygiene Rating Scheme in which commercial food establishments are inspected and scored with the results made public. In this study we investigate the prevalence of food risk increasing behaviours among chefs, catering students and the public. Given the incentive for respondents to misreport when asked about illegal or illicit behaviours we employed a Randomised Response Technique designed to elicit more accurate prevalence rates of such behaviours. We found 14% of the public not always hand-washing immediately after handling raw meat, poultry or fish; 32% of chefs and catering students had worked within 48 hours of suffering from diarrhoea or vomiting. 22% of the public admitted having served meat “on the turn” and 33% of chefs and catering students admitted working in kitchens where such meat was served; 12% of the public and 16% of chefs and catering students admitted having served chicken at a barbeque when not totally sure it was fully cooked. Chefs in fine-dining establishment were less likely to wash their hands after handling meat and fish and those who worked in award winning restaurants were more likely to have returned to work within 48 hours of suffering from diarrhoea and vomiting. We found no correlation between the price of a meal in an establishment, nor its Food Hygiene Rating Score, and the likelihood of any of the food malpractices occurring.

## Introduction

There are an estimated 500,000 cases of foodborne disease linked to known pathogens in the UK annually [1], and 9.4 million in the US [2]. Associated with these illnesses are medical, financial and welfare costs, estimated to be £1.8 and $14 billion respectively [3, 4].

A large proportion of foodborne illness in the UK is considered avoidable [5]. While much investment and research is focused on making foods safer in early stages of the food chain, for example by vaccination (e.g. *Salmonella* in eggs), the role of food handlers/preparers is still a crucial point of risk and potential intervention [6]. Practices can render previously uncontaminated foods unsafe to eat e.g. through cross-contamination; and contaminated foods safe to eat e.g. through thorough cooking [6, 7]. The latter is particularly important when handling food products that have high contamination rates at the point of retail e.g. the 70% of UK supermarket chickens that are *Campylobacter* positive [8].

Approximately 60% of foodborne disease outbreaks are linked to eating establishments and commercial caterers [9]. Multiple risk factors for foodborne illness are commonly implicated in outbreaks including inadequate heat treatment (50%), inappropriate storage (45%), cross-contamination (39%) and infected food handlers (12%) [10]. Domestic kitchens are also a significant source of sporadic foodborne disease cases [11].

The public have been targeted via information campaigns such as Food Safety Week [5, 12] and the catering industry through inspection and sanction, for example the Food Hygiene Rating Scheme (FHRS) implemented in 2013. A challenge for such campaigns is that knowledge does not always translate to behavioural change of domestic or commercial food handlers [13].

The FHRS inspection regime established by the UK FSA, is a composite score for food handling, physical structure, facilities and how the business manages and records its food safety processes. The score is available to consumers online (http://www.food.gov.uk/business-industry/caterers/hygieneratings) via a smartphone app (http://www.food.gov.uk/about-us/data-and-policies/app) and in establishments’ doors/windows. Display of the FHRS score at premises is mandatory in Wales and the extension of this mandatory regime is under consideration for England. The system differs geographically within the UK. For example, in England, Wales and Northern Ireland, a six-point scale is used, where values 0–2 are considered unacceptable, with 3–5 ranging from satisfactory to very good. The Scottish system is binary, indicating either ‘Pass’ or ‘Improvement Required’.

Such inspections are, by their nature, snapshots and determining the true prevalence of food malpractices is problematic. Research on food handling typically relies on self-reported behaviours, which may be subject to social desirability bias [11]. Misreporting may also be motivated by a desire to avoid embarrassment [14] and in commercial settings, admitting to food safety malpractice can be incriminating. Hence, direct questioning may prompt over-reporting of good, and underreporting of bad, food safety practices [13, 15, 16].

The risk of systematic misreporting has led to the development (in other domains) of questioning techniques which induce greater truth telling and reveal more accurate estimates of the prevalence of sensitive behaviours. Methods such as the Randomised Response Technique (RRT) and the Item Count Technique [14, 17] introduce randomisation or uncertainty into the question-answer process, protecting respondents by obscuring their answer. RRTs use a randomisation device (e.g. dice) to determine how respondents answer a sensitive question [18, 19]. The researcher adjusts the results using the known probabilities of the dice outcomes that prompt a forced answer.

RRT studies in diverse disciplines have generated higher estimated prevalence rates than anonymous direct questioning [20–22]. Validation studies, with access to true rates of the sensitive behaviour, have also shown the superiority of RRT techniques over direct questioning [23, 24]. The forced response model is one of the most statistically efficient RRT designs [19], and is employed here for the first time in determining the prevalence of food handling malpractices.

This study focuses on poor food safety practices in kitchens. It is concerned with rates of Food Risk Increasing Behaviours (FRIBs). Given the importance of both commercial and domestic sectors in the food disease burden, we investigate such behaviours among the public and professional chefs. RRT, designed to more accurately reveal rates of illicit behaviours, was implemented with the objectives of:

1. determining the prevalence of FRIBs amongst working chefs, catering students and the public;
2. investigating whether food malpractices are correlated with observable characteristics among the general public (gender, age, attitudes to risk, etc);
3. investigating whether food malpractices are more likely in certain types of commercial establishments (FHRS score, price band, awards won) and correlated with observable characteristics of chefs and catering students (gender, position etc);
4. exploring the implications of the prevalence of poor practices for food hygiene and human health.

## Materials and methods

### Survey design: Selection of food risk increasing behaviours

We selected four Food Risk Increasing Behaviours (FRIBs) for investigation using RRT. Noting that meat “on the turn” is a colloquial expression referring to meat (fresh or raw) that is no longer fresh, something which will be apparent from its smell and possibly taste, the four behavioural statements presented to chefs and catering students were:

1. I always wash my hands immediately after handling raw meat, poultry or fish
2. I have worked in a kitchen within 48 hours of suffering from diarrhoea and/or vomiting
3. I have worked in a kitchen where meat that is ‘on the turn’ has been served
4. I have served chicken at a barbeque when I wasn’t totally sure that it was fully cooked

The four behavioural statements presented to the public were:

1. I always wash my hands immediately after handling raw meat, poultry or fish
2. I have cooked food for others within 48 hours of suffering from diarrhoea and/or vomiting
3. I have served meat that is ‘on the turn’
4. I have served chicken at a barbeque when I wasn’t totally sure that it was fully cooked

Behaviours 1 and 2 relate to food hygiene basics and should feature in (the prerequisite programs of) the businesses’ HACCP. These behaviours have the potential to contaminate food with bacteria and represent two extremes of HACCP failing. The need for good hand hygiene is likely to be the most commonly communicated food hygiene message and should therefore be simple and accessible to respondents, whilst working within 48 hours of suffering from diarrhoea and/or vomiting contravenes UK regulations which state that “m*anagers must exclude staff with these symptoms from working with or around open food*, *normally for 48 hours from when symptoms stop naturally”* [25]. For the public, washing hands is easily achievable, and well known good practice.

Behaviour 3 relates to serving meat that is spoiling, and is a previously unexplored behaviour suspected of being practised in some catering establishments (discussed later in the paper) which has potential implications for foodborne illness.

Behaviours 2 and 3 were of interest because these are unlikely to be identified by direct observation of kitchen behaviours or an inspection. Behaviour 2 was also selected as it was identified as a significant issue in one of the highest profile outbreaks of food poisoning in recent years in the UK, in which over 400 diners fell ill after eating at the Michelin-starred restaurant “The Fat Duck” (a case discussed later in the paper) and has been identified as a factor in other outbreaks [26].

Behaviour 4 was selected for investigation because undercooked chicken and barbecued meat are known risk factors for campylobacteriosis [1, 27–29] the most commonly reported gastrointestinal bacterial pathogen in humans in the EU since 2005 [30]. Handling, preparation and consumption of broiler meat may account for 20% to 30% of human cases of campylobacteriosis, while 50% to 80% may be attributed to the chicken reservoir as a whole [31, 32]. A notable feature of the profile of campylobacter cases is its seasonality, with a ‘spring peak’ identified consistently [33, 34]. Barbecuing might contribute to this seasonality [28, 35–37] and is increasingly widespread. In 2010 there were over 120 million barbecue events in the UK [38]. An additional motivation for including behaviour 4 was that barbecuing, and the cooking of chicken in general, has been the focus of repeated FSA campaigns aiming to reduce the number of chicken-related Campylobacter cases. These have included the 2014 “Don’t Wash Raw Chicken” campaign and 2015’s campaign entitled “the Chicken Challenge” (#ChickenChallenge) aimed at helping cut campylobacter food poisoning in half by the end of 2015.

### Survey design: Randomised response protocol

Various RRT approaches have been employed in the literature. We used the forced response RRT, attributed to Boruch [39], with respect to the four food behaviour statements listed above. Respondents were asked to roll two dice. They were then asked to answer the sensitive question following these instructions:

- Add up the numbers on the two dice
- If they add up to 2, 3 or 4, always answer Yes (regardless of your true answer)
- If they add up to 5, 6, 7, 8, 9 or 10 answer the question truthfully
- If they add up to 11 or 12, always answer No (regardless of your true answer)

Each statement was presented separately with “Yes” and “No” answer tick boxes, and respondents were reminded to roll the dice again and follow the instructions for each question. Only the interviewee knew the outcome of the dice roll. The interviewer was thus unable to distinguish an answer forced by the dice roll from an admission of the sensitive behaviour. This ensured both respondent privacy and protected the interviewer from being aware of potential malpractice.

Based on the probability of dice rolls, the proportion of respondents theoretically instructed to answer yes is known (1/6), as is the proportion instructed to answer truthfully (3/4). This technique allows the prevalence of true bad behaviours in the sample to be estimated but precludes determination of any individual’s behaviour.

To promote compliance with RRT instructions we followed the recommendations of Lensvelt-Mulders and Boeije [40] for successful RRT implementation including acknowledging to respondents that being “forced” to answer contrary to the truth is difficult but explaining that this is necessary for the technique to succeed, and explaining to the respondents how they were protected to increase the rate of compliance with the protocol.

### Data collection

Four target groups were identified for sampling: chefs, catering students with restaurant experience, catering students without restaurant experience and the public. A questionnaire was designed for each sample, retaining as much commonality as possible but reflecting the differences between them. Each of the surveys featured four RRT behavioural statements, worded to suit the respondent group.

Each group was asked a set of additional questions on characteristics which may help to explain their food hygiene behaviours. For chefs and working students these included questions on: kitchen position, the type of restaurant they work in, average price of a main meal, food hygiene rating score and whether their kitchen had won awards or accolades. Members of the public were asked about their experience of food poisoning, their level of concern about food poisoning and their cooking role at home. Demographic information (age, gender, education level etc.) was collected from all respondents.

The public sample (N = 926) was recruited via an online market research panel (ResearchNow). The chef sample (N = 132) was recruited through face-to-face convenience sampling at culinary shows and competitions and via online culinary forums. Catering students were recruited through pre-arranged college visits and at culinary shows and competitions, giving a sample of 61 students with commercial experience, and 45 without.

All face to face sampling required the interviewer to explain and demonstrate the RRT technique and rationale. The respondent rolled the dice in an opaque beaker to ensure privacy. Online surveys featured an embedded screencast explaining the RRT technique and rationale with a pair of virtual dice appearing in a pop-up window from a 3^rd^ party website (to further reassure respondents that the die rolls were not being recorded by the researchers).

Data were collected in England, Wales and Scotland in 2014 and 2015. Informed consent was obtained from all participants: chefs/ students signed a consent form, the online public sample completed a consent check list before proceeding with the survey. Participants were debriefed on the purpose of the survey after completion, and given the opportunity to withdraw their data. Ethical approval was obtained from the College of Natural Science Ethics Committee at Bangor University, reference number CNS/2014/AJ1.

### Data analysis

To determine the prevalence rates of the FRIBs, the response data required adjustment, given the randomisation protocol. This employed the known probabilities of people giving ‘false’ yes and no answers.

Given the structure of the forced choice question, the probability that individual i gives a ‘yes’ response is given by:

$$P(y_{i})=\pi_{1}+(1-\pi_{1}-\pi_{2})P(Y_{i})$$ (1)

Where

y = reported behaviour, y = 1 for yes, 0 for no

Y = true behaviour, Y = 1 for yes, 0 for no

*π*_1_ = probability that a respondent is instructed to answer ‘yes’

*π*_2_ = probability that a respondent is instructed to answer ‘no’

It is possible to estimate the true proportion in the sample exhibiting the behaviour from:

$$\overset{⌢}{Y}=\frac{\overset{⌢}{y}-\pi_{1}}{1-\pi_{1}-\pi_{2}}$$ (2)

Where

$\overset{⌢}{y}$ = the observed fraction reporting an answer of ‘yes’ [17].

The variance of the estimated prevalence rate is given by

$$\text{var}(\overset{⌢}{Y})=\frac{\overset{⌢}{y}(1-\overset{⌢}{y})}{n\times {\left(1-\pi_{1}-\pi_{2}\right)}^{2}}$$ (3)

Where:

*n* = total number of respondents

This exposition is for the case where a ‘Yes’ answer indicates a FRIB. For Question 1, where a “No” implies a FRIB, the definition of y and the forcing probabilities are redefined appropriately. The standard error (SE) was taken to be the square root of the calculated variance and the 95% confidence intervals as the prevalence rate ± 1.96 SE [17].

It is possible to identify if individual specific characteristics influence the probability of FRIBs, even if responses are masked by the RRT technique, using an extension of the standard logit model. The probability that an individual response will be a ‘yes’ is given by:

$$P(y_{i})=\pi_{1}+(1-\pi_{1}-\pi_{2})\frac{\text{exp}(\beta X_{i})}{1+\text{exp}(\beta X_{i})}$$ (4)

Where X_i_ are a set of individual specific determinants that may influence the true underlying behaviour [41]. The model is estimated as a multiple regression with a vector of explanatory variables using the rrlogit command (v1.1.2) [42] in Stata 13.1.

Explanatory variables tested included characteristics of the person (chefs, public) and their employment status and type of institution in which they worked (chefs). For the public sample the characteristics tested were age, gender, university education and social class (defined as A, B or C1 as opposed to C2, D or E where A = upper middle class; B = middle class; C1 = lower middle class, as opposed to C2 = skilled working class; D = working class; E = non-working). Attitudes and perceptions tested were whether they considered themselves to be ‘adventurous when eating out’, how concerned they were about food safety at home and their perceived risk of getting food poisoning compared with other people. The coding of these variables is shown in Table 1.

**Table 1:** Summary statistics for public sample (n = 905^†^).

Variable	coding/units	Sample mean
Adventurous^$^	likert 1–5	3.1
Female	yes = 1; no = 0	0.56
University education	yes = 1; no = 0	0.34
Concern at home^#^	likert 1–4	2.4
Risk^^^	likert 1–5	2.5
Social class A,B,C1	yes = 1; no = 0	0.60
Age	years	45.5

^†^926 answered the RRT questions but not all of these answered the demographic / explanatory questions

^$^Adventurous when eating out: strongly disagree (1) disagree (2) neither (3), agree (4), strongly agree (5)

^#^ Concerned about food safety at home: not at all (1) slightly (2) moderate (3) very (4)

^Compared with other people my risk of getting food poisoning: much less (1) less (2) same (3) more (4) much more (5).

Additional variables tested for the chef sample were working status, number of years worked, price band of their employing establishment and whether that establishment: was a fine dining establishment; had won awards; had passed a food hygiene inspection. The coding of these variables is shown in Table 2.

**Table 2:** Summary statistics for chef sample.

Variable	n	coding/units	Sample mean
Chefs	237	yes = 1, no = 0	0.55
Working Students	237	yes = 1, no = 0	0.26
Non-working students	237	yes = 1, no = 0	0.19
Time Worked	237	years	9.1
Age	235	years	31.4
Female	236	yes = 1; no = 0	0.25
Fine dining	193^$^	yes = 1; no = 0	0.30
Award	193^$^	yes = 1; no = 0	0.24
FHRS_pass	193^$^	yes = 1; no = 0	0.79
Main Meal Cost	124^#^	£s	13.35

^$^Chefs and working students only

^#^Chefs only

The coding of the variable concerning food hygiene inspection status requires some explanation.

The hygiene scoring system differs between England/Wales and Scotland. These scores were manipulated and combined to generate a dummy (0,1) variable (FHRS_pass). A “satisfactory performance” value of 1 was assigned to establishments in England/Wales with Food Hygiene Rating Scheme (FHRS) scores of 3–5 and those from Scotland which had a “pass” score. The alternative category (FHRS_pass = 0) combined those who held an unsatisfactory score (FHRS score of 0–2 in England/Wales or an ‘Improvement Required’ score in Scotland).

Interpretation of the magnitude of the estimated coefficients in the logit model in (4) is somewhat opaque. More intuition is provided by the estimated marginal effects, defined as the change in probability that arises from a marginal change in an attribute. The nonlinearity of the logit model means that the marginal effects vary across the response surface. We calculate the marginal effects at the probability evaluated at the mean of the independent variables. For a continuous variable this is:

$$\frac{\partial P(y)}{\partial X}=\bar{p}(1-\bar{p})\beta$$ (5)

where $\bar{p}$ is the probability of answering yes, evaluated at the mean of all exogenous variables.

For categorical variables (for example a 0,1 ‘dummy variable’ defining gender etc) we report the discrete first difference for the probabilities when the variable = 0 and = 1. Standard errors and the significance of the marginal effects are derived from the logit parameter estimates.

It is also possible to predict individual specific probabilities that an individual will commit a FRIB, for all individuals in the sample, based on the parameter estimates derived from model (4), and their personal characteristics (*X*):

$$P({\hat{Y}}_{i})=\frac{\text{exp}(\hat{\beta }X_{i})}{1+\text{exp}(\hat{\beta }X_{i})}$$ (6)

Such an analysis combines the estimates of the impact of attributes on behaviour with their prevalence in the sample and, in particular, their co-occurrence in the sample.

## Results

### Sample characteristics

Tables 1 and 2 report the summary statistics for the samples.

### Food risk increasing behaviours: Public

Table 3 reports the estimated prevalence rates of the four behaviours among the public, with associated standard deviations following Petroczi, Nepusz [17].

**Table 3:** Inferred prevalence rates of risk increasing behaviours among the public (n = 926).

	Prevalence	s.d.
Not hand washing	13.7	1.5
Served meat “on the turn”	22.0	1.8
Cooked for others within 48 hours of diarrhoea and vomiting	29.3	2.0
Served chicken at barbecue when not sure it was fully cooked	12.8	1.5

Estimation of the logit models in (4) provides estimated coefficients and marginal effects, which are shown in Table 4. The results indicate that, *inter alia*, the probability of serving meat on the turn was 11 percentage points higher for those with a University education. University graduates were also more likely to have worked within 48 hours of experiencing diarrhoea and vomiting (9 percentage points), as were those who believed they were more at risk of food poisoning than the average person (9 percentage points). Those who considered themselves as adventurous when eating out were more likely to have served barbeque chicken when not sure it was cooked (3.5 percentage points) whilst women were significantly less likely to have done so (8 percentage points).

**Table 4:** Estimates of extended logit and marginal effects of attributes on probability of bad behaviours: Public sample.

		Not hand washing	Served Meat ‘on the turn’	Working within 48h of D&V	Served chicken when unsure if cooked
Respondent characteristics:					
Adventurous	coefficient	-0.041	0.219*	0.026	0.348*
	marginal effect	-0.5	3.7*	0.5	3.5**
Female^$^	coefficient	0.025	-0.243	0.184	-0.786**
	marginal effect	0.3	-4.1	3.7	-8.3**
University education^$^	coefficient	0.259	0.619**	0.434**	0.194
	marginal effect	3.0	11.0**	9.1**	2.0
Concern at home	coefficient	-0.409***	-0.062	-0.019	-0.226
	marginal effect	-4.5***	-1.0	-0.4	-2.3
Risk	coefficient	0.057	0.052	0.434***	-0.083
	marginal effect	0.6	0.9	8.9***	-0.8
Constant		-1.058	-2.032***	-2.292	-1.993
Log Likelihood n		-426.73 905	-570.17 905	-597.74 905	-514.29 905

Marginal effects in parentheses: percentage point change in the probability of a FRIB given a marginal change in attribute.

^$^Indicate dummy (0,1) variables

*,**,*** indicate P>|z| <0.1,0.05,0.01 respectively

The marginal effects reported in Table 4 show systematic effects of characteristics of person or employing institution on the probability of a FRIB being committed. Additional insights regarding the degree of variation in those probabilities is conveyed in Fig 1 which shows the distribution of simulated, individual level, probabilities derived from (6).

**Fig 1:** Distributions of members of the public’s (n = 926) simulated probabilities of committing the four studied food risk increasing behaviours.

The relatively low power of the models in predicting behaviour is manifested in the concentration of the values around the sample means, and the absence of groups with a particularly high predicted probability of performing the behaviour. However, these distributions do show the extent to which the model can differentiate among individuals on the basis of their characteristics.

### Food risk increasing behaviours: Chefs and catering students

Table 5 reports the estimated prevalence rates of the four behaviours among chefs and catering students, with associated standard deviations derived following Petroczi, Nepusz [17].

**Table 5:** Prevalence rates of four typical bad behaviours amongst chefs and catering students.

	Prevalence	sd
Not hand washing (n = 238)	7.4	2.2
Meat served on the turn (n = 193)^$^	33.0	4.5
Working within 48 hours of diarrhoea and vomiting (n = 238)	31.6	4.0
Served barbeque chicken when not sure fully cooked (n = 203)^#^	15.9	3.4

^$^ non-working students were not asked this question

^#^ this question was added to the survey after initial piloting, so the sample is reduced.

A third of the sample had worked in kitchens where meat on the turn was served. Almost one third (32%) reported working in a kitchen within 48 hours of suffering from diarrhoea and/or vomiting. The proportion of chefs and catering students not hand-washing immediately after handling raw meat, poultry or fish was about half that of the public sample at 7.4%.

An understanding of the type of person and/or establishment in which behaviour such as working within 48 hours of experiencing D&V or serving meat on the turn was most likely to occur is of interest both from a regulatory point of view but also from the perspective of consumers wishing to reduce their risk of exposure to food prepared in such conditions. Table 6 reports estimates of coefficients and marginal effects. The first model uses characteristics of the individuals, the second model uses characteristics of the establishment they work in.

**Table 6:** Estimates of extended logit and marginal effects of attributes on probability of bad behaviours: Chef and catering student sample.

		Not hand washing	Meat ‘on the turn’ Served ^Φ^	Working within 48h of D&V	Served chicken when unsure if cooked
Respondent characteristics:					
Working student^$^	coefficient	-1.385	-0.595	-0.763	0.244
	marginal effect	-5.5	-12.5	-15.2	0.8
Non-Working Student^$^	coefficient	-0.720		-0.828	-15.797***
	marginal effect	-3.1		-15.9	-19.0***
Head chef^$^	coefficient	-1.767	-1.232**	-0.114	-0.622
	marginal effect	7.2	-25.0**	-2.4	-1.7
Time	coefficient	-0.035	0.014	-0.014	-0.007
	marginal effect	-0.00	0.3	-0.3	-0.0
Constant		-1.519*	-0.242	-0.261	-1.223*
Log likelihood value		-94.86	-127.81	-158.89	-118.36
n		237	192	237	203
Establishment characteristics:					
Fine dining^ψ^	coefficient	2.900	0.228	0.029	-0.252
	marginal effect	18.0*	5.0	0.6	-3.7
Award^ψ^	coefficient	0.416	-0.726	1.199**	0.443
	marginal effect	1.4	-14.8	27.8**	7.3
FHRS_pass^ψ^	coefficient	0.092	-0.024	-0.172	0.496
	marginal effect	0.3	-0.5	-3.8	6.9
Constant		-4.503*	-0.595	-0.909*	-1.871**
Log Likelihood		-72.47	-130.13	-127.65	-109.34
n		193	193	193	177

Marginal effects in parentheses: percentage point change in the probability of a FRIB given a marginal change in attribute.

^$^Indicate dummy (0,1) variables

^ψ^Indicate dummy (0,1) variables

^Φ^ this question was not asked of non-working students

*,**,*** indicate P>|z| <0.1, 0.05, 0.01 respectively

There were no systematic effects predicting the probability of all four risk-increasing behaviours, but there were individual effects. Working in a fine-dining establishment increased the probability of not washing hands after handling meat and fish by 18 percentage points. Chefs and students who worked in a restaurant that had received an accolade or award were more likely to have returned to work within 48 hours of suffering from diarrhoea and vomiting (28 percentage points). We found no correlation between the price of a meal in an establishment and the likelihood of FRIBs occurring—despite over a third of the public sample (36%) agreeing that the more expensive a meal was the safer they would expect it to be. Furthermore there was no relationship between an establishment having an unsatisfactory FHRS score and rates of any of their FRIBs occurring. This suggests that chefs from establishments rated as ‘satisfactory’ are as likely to engage in bad behaviours as those rated ‘unsatisfactory’.

There is no evidence of a lower prevalence of risk-increasing behaviours in more expensive, award-winning or fine-dining establishments. Where significant effects occurred, they suggested the reverse: higher rates of poor hand-washing in fine-dining establishments and chefs in award winning kitchens more likely to return to work too soon after an episode of diarrhoea and/or vomiting. Perhaps most notable of all is the absence of a relationship between the probability of FRIBs occurring and the chef’s establishment having an (un)satisfactory FHRS score.

## Discussion

Food behaviours, in both domestic and commercial kitchens, have the potential to create or exacerbate food safety hazards. The prevalence of illicit, food risk increasing behaviours are difficult to determine via direct questioning and observational studies, given their sensitive and often fleeting nature. In this study a forced response RRT technique, proven to improve estimates of illicit or embarrassing behaviours in other fields, was employed to estimate the prevalence of four FRIBs.

### Methodological considerations

There is considerable evidence that RRT provides more accurate estimates of sensitive behaviours compared to direct questioning survey methods [18]. However, due to the inherent noise associated with forced response approaches, RRT requires larger samples compared to conventional techniques in order to obtain estimates with acceptable levels of error [43, 44]. Larger sample sizes require a contingent increase in research costs. However, it is suggested that increased costs are compensated for by the corresponding increase in data validity [19].

Whilst this method seeks to reduce the impact of social desirability bias it does not, however, account for the desire to reduce cognitive dissonance (the mental discomfort felt when knowledge and behaviour differ) and inaccurate memory formation and recall. These factors may partially account for the higher than expected rates of handwashing we report [45]. The similarity between the handwashing rates in this study and from comparable direct questioning studies suggest that these factors could be more important in the underreporting of poor hand hygiene behaviours than the social desirability bias controlled for by RRT. The RRT is therefore suggested as a useful means of determining the prevalence of sensitive, non-routine food behaviours, where social desirability bias is thought to be a primary reason for misreporting.

### Prevalence of food risk increasing behaviours

The proportion of chefs and catering students identified as not hand-washing immediately after handling raw meat, poultry or fish was 7.4%. Rates of poor hand washing practice were higher among the public than the chef and student sample. Both estimates are comparable to rates obtained from direct questioning studies in the UK and Ireland e.g. 6% from face to face interviews with 200 Irish chefs [46] and 14% amongst the public from the Food Standards Agency’s large scale *Food and You* study [47]. Far higher rates have been reported in other studies e.g. 23% amongst chefs (based on telephone direct questioning) in a US study by Green and Selman [48] and 47% to 100% in observational studies in the UK, USA and Australia [11, 49–51].

It is of serious concern that almost one third of the surveyed chefs and students reported working in a kitchen within 48 hours of suffering from these illnesses. There is no comparative previous UK figure for this behaviour, however the rate is higher than those identified in US studies (using face to face or telephone questioning) where rates of between 5% and 20% were reported by Carpenter, Green [52], Sumner, Brown [53] and Green, Selman [16]. The lower rates recorded in the US may result from better hygiene practices, the acute sensitivity of admitting this behaviour in response to direct questioning, or a combination of the two. In the UK such behaviour contravenes Food Hygiene Regulations, which state that:

“*No person suffering from*, *or being a carrier of a disease likely to be transmitted through food or afflicted*, *for example*, *with infected wounds*, *skin infections*, *sores or diarrhoea is to be permitted to handle food or enter any food-handling area in any capacity if there is any likelihood of direct or indirect contamination*” [54]. Managers are required to exclude staff with symptoms such as diarrhoea and vomiting from working with or around open food, normally for 48 hours from when symptoms stop naturally.

Such risk increasing behaviour is not solely confined to “low-end” restaurants. Staff working too soon after illness, and hence still infectious, was a factor cited in the investigations of the outbreak of food poisoning at Michelin-starred chef Heston Blumenthal’s Fat Duck restaurant in 2009 [55]. The Health Protection Agency (HPA) criticised practices at the restaurant in its investigations after over 500 of the restaurant’s customers fell ill. The HPA later detected norovirus infection in six staff and reported that "*Based on staff interviews*, *sickness records and samples taken*, *it is clear that staff worked while still infectious with norovirus*,” [55]. Of the staff interviewed, 17 reported having had symptoms of gastrointestinal infection in the period under investigation of whom six reported working while unwell, including one who reported vomiting in the restaurant toilets. Nine staff reported returning to work before being asymptomatic for 48 hours.

The rates of serving of food within 48 hours of an episode of diarrhoea and vomiting are similar for the public at about 30%. However, the legal and wider food safety implications of such behaviour are different for chefs than for those at home. For the latter there may often be no feasible alternative to them preparing food shortly after illness, particularly if there are children in the household.

The high proportion of chefs and students admitting to having worked in a kitchen where meat ‘on the turn’ has been served is also of concern for public health. There are no comparative rates of this behaviour in other studies, although the practice is a long-established means of reducing costs in restaurants. Chefs interviewed for a UK television programme on ‘kitchen confessions’ explained that “*the first task we gave someone who came to us looking for a cheffing job was to make a meal with the chicken that was 'on the turn' … That's important to a kitchen because it means you can get another day or two days out of your meat*. *If a chef could do this I knew he was experienced in restaurant kitchens"* [56]. The use of rich, heavy sauces was cited by another who reported having *"worked at a place where we served steak and chips on a Saturday a 'special value' steak on Sunday and a steak in a spicy pepper sauce on Monday*. *By that point the meat…was almost inedible but we'd mask it with a heavily flavoured sauce rather than bin it*.*"*

Interest in the rate of serving undercooked chicken at barbecues was motivated by the current UK policy focus on *Campylobacter* and the argument that barbecues may contribute to the annual ‘spring peak’ identified in campylobacter cases. These factors led the FSA to denote *Campylobacter* as their priority pathogen (alongside *Listeria*) in the 2010–2015 Foodborne Disease Strategy [5] and educational campaigns centred around safe barbecuing and the safe cooking of chicken in 2014 and 2015 respectively. The rate of serving chicken at barbecues when unsure it was fully cooked was higher among the chefs and catering students than the public (16% versus 13%) contrary to the expectation that the professionally trained would be less prone to this behaviour. The frequency with which barbecues are held, the popularity of serving chicken at them, the high rates of contaminated chicken sold in the UK (c.70% in 2015) and the role of undercooked chicken as a Campylobacter risk factor, means this behaviour represents a serious public health problem in the UK.

### Implications of our findings

This study suggests that behaviours that may be important risk factors for foodborne disease are widely prevalent and likely to be missed by direct observation studies and restaurant inspections. There are likely to be varied and multiple causal factors behind the behaviours. A lack of time, staff and resources are consistently identified as barriers to compliance with safe food procedures such as handwashing [13, 48, 57]. There is a clear economic imperative to serve meat “on the turn” and existing behavioural norms within commercial kitchens will affect new members of staff employed within them. The motives leading to workers opting to (return to) work whilst still posing risk of transmission after illness is multifaceted. Ignorance, the economic losses associated with not working, fear of losing one’s job and the desire not to let down colleagues (or the family business) are all possible causes of the behaviour [52].

Regardless of the causes, the prevalence of such behaviours is problematic for consumers. When dining out consumers use a variety of information sources and heuristics to make choices. They may believe that they are less vulnerable to food risk increasing behaviours when they opt to dine at a ‘fine dining’ restaurant, one with awards and where prices are higher and the FHRS score is good. For the FRIBs we considered, those assumptions and heuristics were unsupported. Where significant effects were identified (see Table 6) they were contrary to what might be plausibly expected: poor hand washing was more common among chefs working in “fine dining” establishments, working within 48 hours of diarrhoea and vomiting occurred more often in award winning restaurants. Neither the price band of the establishment, nor its FHRS score, had an effect on the probabilities of the FRIBs.

The FSA has established the FHRS as a means to help the public “choose where to eat out …by telling you how seriously the business takes their food hygiene standards” [58]. The results presented here are not a systematic evaluation of the FHRS. However, the lack of an effect of an (un)satisfactory FHRS on the rate of the FRIBs sounds a note of caution. These results in combination suggest that the challenges for the public in finding outlets serving safer food continue to be considerable, with many of the cues they might refer to, and heuristics they might employ, being of limited help.
